The article "Immersive Learning Method of Ideological and Political Education under Big Data and Artificial Intelligence" was retracted in 2023. Reasons: unreliable results or conclusions; concerns about the data; concerns about the peer review; concerns about the citations.

# Immersive Learning Method of Ideological and Political Education under Big Data and Artificial Intelligence

**DOI:** 10.1155/2022/4176595

**Published:** 2022-06-15

**Authors:** Yan Yu

**Affiliations:** School of Marxism, Beijing Information Science & Technology University, Beijing 100192, China

## Abstract

The study aims to explore the influence of big data on college students' learning methods of ideological and political education (IPE) under artificial intelligence. First, the characteristics of big data are analyzed. Second, big data is introduced into IPE's classroom teaching, and its influence on students' learning methods is discussed. Finally, the questionnaire is designed to investigate students' learning attitudes and teachers' effectiveness. The results show that the scores of the students are poor, and the traditional teaching method should be updated to improve the teaching quality of IPE. Motivating students' enthusiasm and updating the teaching content are the main tasks to improve students' learning effect on IPE. College students who receive IPE based on big data have better academic performance and a positive learning attitude, and each factor is more significant than 0.05. It is concluded that big data has a considerable impact on IPE. It can promote students' mastery of the knowledge and improve their learning efficiency.

## 1. Introduction

With the progress of society, new requirements have been put forward to the teaching quality of ideological and political education (IPE) in colleges. General Secretary Xi Jinping proposes to use big data to optimize IPE and promote the innovative development of college students under artificial intelligence (AI). The application of network media and data analysis technology changes students' thinking mode and teachers' teaching methods and resources, forming a new background of IPE [1]. According to the survey, the college students' WeChat usage rate is 100%, and short videos are increasingly common. Students can get information from similar we-media platforms and express their attitudes via “likes,” “comments,” or “forwarding” [2]. Students who hold the same views are often affected by the cluster effect and gradually form a group. In the ideological and political theory class, they often conflict with the public's attitude because of their own attitude. Therefore, college IPE teachers must fully understand students' attitudes towards specific events and problems. Otherwise, it is difficult for students to have feelings in the learning process to make the contents learned really enter the brain and heart. Teachers should always optimize and adjust the teaching contents according to students' needs and social changes in the teaching process. In teaching the IPE theory in the classroom, teachers should combine the hot spots of public social opinion into the teaching through their own analysis, making the IPE classroom a modern classroom that truly conforms to the development of the times [3]. As Internet natives, college students tend to search for diversified expressions to meet their personalized needs. Under global intervention of data analysis and intelligent computing technology, IPE is deeply embedded with science and technology in the practice, theory, and logic to realize technical transformation. Big data can reflect the large-scale social changes at the beginning of the twenty-first century. Big data and information processing realize the real-time acquisition and classification of students' overall information and ideological and behavioral changes and facilitate the renewal and innovation of the teaching content of IPE. The data acquisition method creates a high-capacity network information environment to improve the traditional teaching mode. The enormous amount of information carried by the Internet includes the excellent traditional culture, the latest social trend, the best scientific and technological achievements, and the daily updated network public opinions. It becomes the commonly used information resource database for students inside and outside the classroom. Due to the freedom of the information acquisition mode and imperfect network accountability mechanism, more and more disadvantages of the traditional teaching mode appear. Therefore, big data is used to improve the teaching quality of IPE, which has great significance in improving the current situation of IPE.

This work aims to study immersive ideological and political learning through big data technology under the background of AI. The experimental group is set. The students who accept the ideological and political teaching mode under big data technology in the experimental group are studied and compared with the control group. The research innovation is the pretest and posttest of the experimental and control groups, respectively, making the experimental data more accurate and the conclusion more convincing. This work will also provide a reference for applying big data technology in college teaching in the future.

## 2. Related Work

AI technology has been used in all walks of life with its continuous progress. Among them, some research teams conducted investigation and research on the use of AI technology in the education industry.

Yang et al. established a classroom model of the rain mechanism. Without changing the original optimization method, this mechanism randomly initialized several model parameter combinations (submodels) and allowed them to search parameters according to their own optimization methods. At a certain interval of iterations, all submodels were called to the submodel parameter combination with the lowest loss function value, covering three stages of the teaching process: before, in, and after class. Next, the model was applied to the film and television appreciation course, and the key problems in each stage were described. The results show that rain classrooms can significantly improve the learning effect of the target course in all aspects. The participation of big data technology in teaching makes students more attentive. Students can actively participate in group activities and confidently state their findings [4]. Park puts big data technology and digital technology into use in students' teaching. The results show that the introduction of this technology can adjust the focus of educational institutions to better meet students' needs and make students' learning enthusiasm higher [5]. Sergeeva et al. designed and implemented a new set of AI simulation courses to help teachers choose better teaching methods for educating students of different majors. The results reveal that positive teaching methods should be given priority in secondary vocational education institutions. It will increase students' learning activities, promote the development of their initiative and personal potential, produce their creative methods, and solve important teaching and organizational tasks. The investment of AI imitation teaching method makes teachers realize their potential in improving their teaching level by implementing the model of competitive experts in the process of education [6].

The above-related research reveals that AI technology applied to education is gradually maturing. Among them, the classroom model of rain mechanism is more suitable for the current actual teaching, but it cannot obtain and utilize the external teaching resources in real-time and efficiently. This work expects to study students' learning experience and analyze teachers' teaching effect after the practical application of AI technology + big data technology in teaching.

## 3. Materials and Methods

### 3.1. Features of Big Data

Figure 1 shows the characteristics of big data.

Four aspects of big data-related achievements have been made. One of the characteristics of big data is “having a high value,” which is manifested in data extraction from big data. The research value of big data is enhanced by improving the efficiency of data analysis, transforming low-level into high-level information [7, 8]. The second characteristic of big data is “diversity,” making big data more diverse in forms and types. It covers the following categories: reality and virtual, dynamic and static, and structural and unstructured [9], making a single form of data diversified. The third characteristic of big data is “fast speed,” making the data transmission speed faster. The fourth characteristic is “large capacity,” making the system collect data more extensively [10–12].

Big data affect people's daily life. In response to the higher requirements, many research teams advocate putting big data into colleges' classroom teaching to overcome the disadvantages of the traditional teaching mode [13, 14]. First, big data can stimulate students' learning potential and transform students' thinking. Students can select the data they need from massive data, giving them a sense of autonomy, and their independent ability can be improved. Second, when they face the decadent data, their values will be affected, resulting in distorted value orientation disorder and choice confusion. The teacher's teaching ability also affects data dissemination, variety, and environment [15]. Teachers have changed from the previous “education restriction pattern” to the “two-way interaction pattern” between students and teachers in the classroom.

In the era of big data, intelligent IPE in colleges is an inevitable trend for developing accurate college IPE. Liu pointed out that moving from precision to intelligence is due to the fundamental trend of IPE innovation and development supported by cutting-edge technologies such as big data. It is the demand of the times and the inevitable choice to cultivate new people of the times. In the era of big data, the rich connotation of intelligent IPE in colleges contains the intelligent concept of accurate IPE. First, it emphasizes taking accurate orientation as the logical starting point. Through big data technology, teachers fully collect educators' educational information, discover learners' confusion in the learning process according to the systematic intelligent analysis, and integrate learners' cognitive habits, ability and literacy, knowledge reserve, and thinking characteristics. Then, they comprehensively analyze the overall operation of educational activities by using relevant thinking and aim at problems to adjust educational objectives dynamically in real-time. Second, it emphasizes the core focus on accurate teaching. Based on the personalized sample analysis of students, teachers build students' exclusive learning modeling, accurately analyze the educational objects, push high-quality teaching resources, select the best teaching content, and adjust the teaching methods. Finally, it is emphasized to take accurate evaluation as the foothold. Advanced technologies such as big data collection, analysis, and mining are adopted to continuously collect massive educational data information of learners or teachers and obtain learning reports or teaching reports through data visualization technology. It can scientifically and comprehensively evaluate students' learning effects or teachers' teaching effects. Based on this, more targeted development suggestions are put forward for students' future learning or teachers' future teaching to promote learning and teaching with evaluation [16].

Therefore, teachers should keep pace with the times, including changing ideas and updating their knowledge reserves. Finally, students' attitude to the teachers' teaching mode is involved because big data has the characteristics of “having a high value,” which is the potential value of big data in the application process. In the AI era, the data in the actual teaching process of IPE are viewed as the primary source to improve students' learning efficiency. Therefore, both teachers and students engaged in educational activities need to adjust their original ideas, integrate the concept perception and characteristics of big data, and have a correct attitude towards IPE [17].

### 3.2. Application of Big Data to IPE

Massive data are generated with the popularization of multimedia communication channels. Big data also symbolize the competitive ability of national science and technology. It promotes the decision-making mode change, proving that data determine success or failure [18, 19]. The application of big data increases the number of information dissemination carriers and provides users with more options and data potential in the practical application process. Exploring social relations and competitive modes from the traditional thinking mode to Internet technology is close to human life and makes technology the decision-making role [20]. Data-driven decision-making is a logical induction of objective things, and it can truly reflect the state and change of items. It is more accurate than traditional decision-making, and results are more objective and scientific [21].  Figure 2 shows the data-driven decision-making structure of big data.

Big data-driven decision-making affects the government decision-making and economic development trend at the macro level and significantly impacts medical, health, and education. Under the new situation, it can help promote the data decision-making of IPE from the aspects of the environment, relations, and individual influence [22]. Big data can change the overall teaching environment, create a more diversified and free learning environment for students to freely express their thoughts and opinions, and incorporate the information in various fields into the teaching circle, enriching the diversity of data sources. Big data reshape the relationship between educators and the educated. In the teaching process, the dominant position of students is gradually highlighted, the discourse power is rising progressively, and the teaching management mode is changed into a smooth one. The decision-making scene of education is more complex and changeable, and higher decision-making requirements are put forward. Data analysis suggests that IPE should apply the data-driven decision-making theory [23]. More targeted data need to be mined to establish a data screening, collection, analysis, and output model and rationally use data sources from different channels [24]. Finally, a deeper exploration should be conducted according to the IPE characteristics. The scientificity of data analysis determines the scientificity of the analysis results. Massive data online processing and correlation classification can enhance the intelligence of decision-making. Moreover, the data analysis platform can comprehensively excavate and analyze data, thoroughly understand and use data, cultivate data analysis talents, establish data research paradigm and data analysis database, and promote big data decision-making of IPE.

Zhou et al. found that ideological and political teachers in colleges collected and analyzed relevant information about students' learning and behavior through big data technology, made accurate efforts to students' specific needs, and formulated personalized plans to realize intelligent teaching. Besides, the intelligent learning platform can collect learners' education data in real-time and automatically generate learning reports. Moreover, the platform can intelligently feedback relevant learning information and push corresponding learning resources according to each learner's specific model to realize intelligent learning. In the era of big data, intelligent IPE in colleges perfectly interprets the all-round reform and innovation of big data in the field of IPE in colleges and deeply solves the development problems of traditional IPE [25].

### 3.3. Questionnaire Design and Implementation

#### 3.3.1. Questionnaire Content Design

The questionnaire investigates the influence of big data on college students' immersive learning method and attitude of IPE under AI and teachers' teaching effectiveness after the introduction of big data. The research subjects are 240 students. The experimental group members are the students taught by the big data-based teaching mode, and the control group members are the students taught by the traditional method. The pretest and posttest are taken, and the results are compared. SPSS 25.0 is used to process the questionnaire data.

#### 3.3.2. Reliability and Validity Analysis

The Cronbach's Alpha coefficient is used to analyze the reliability of the questionnaire. Usually, the questionnaire has excellent reliability when the coefficient is above 0.9. It has good reliability when the coefficient is above 0.8. When the coefficient remains above 0.7, the reliability of the questionnaire is qualified and can be used for investigation. Validity analysis is the degree to which the measurement tool makes a measurement. The closer the measurement data are to the standard, the higher the efficiency is. The validity of the questionnaire is tested according to the value of Kaiser–Meyer–Olkin (KMO).

## 4. Statistics and Analysis of the Questionnaire Results

### 4.1. Survey Results Statistics

#### 4.1.1. Gender Distribution of Respondents

Figure 3 shows the statistical analysis of college students' gender in the questionnaire survey.

Figure 3 shows that 168 male students and 72 female students have participated in this questionnaire survey, accounting for 70% and 30%, respectively.

#### 4.1.2. Political Outlook of Respondents

Figure 4 shows the questionnaire's statistical analysis of college students' political outlook.

Figure 4 shows that, among 240 participants, 39 are members of CPC, accounting for 16.3%; the majority of them are members of the Communist Youth League, with a ratio of 75.6%, and 8.1% are masses.

#### 4.1.3. Factors Affecting Teaching Effectiveness

Table 1 shows the statistics of influencing factors of teaching effectiveness.

The data in Table 1 reveal that 80 of the 240 college students who have participated in the survey believe that basic attitudes will impact ideological and political teaching, accounting for about 33.3% of the total. 28.3% of the students hold that the teaching methods of ideological and political teachers will impact the efficiency of students in class. 14.6% of the students believe that the school's ideological and political learning atmosphere will also impact teaching to a certain extent. 23.8% of the students believe that when the content of ideological and political teaching is different, the teaching effect will also change.

#### 4.1.4. Element of Improving the Teaching Quality of IPE

Figure 5 shows the elements of enhancing the teaching quality of IPE.

Figure 5 shows that 85 of the students believe that the teaching mode of IPE needs to be improved. 90 students hold that correct students' learning attitudes should improve the teaching efficiency of IPE. 23 students think that a good learning atmosphere is also one of the factors affecting the teaching quality of IPE. 42 students believe that the teaching method cannot reflect the students' mastery of IPE knowledge. In short, students' academic performance of IPE is poor, and how to motivate students' learning enthusiasm and improve the teaching quality of IPE is the main task to be completed.

### 4.2. Results of Questionnaire Reliability and Validity Analysis

Table 2 shows the reliability test results of the questionnaire.

The test results in Table 2 show that Cronbach's alpha values of all dimensions in the questionnaire are maintained at 0.782–0.927. It shows that the questionnaire has good reliability.  Table 3 shows the validity test results of the questionnaire.

In Table 3, Bartlett's test shows that the approx. Chi-square is 1404.359, and the probability of sig. is 0.000, less than 0.5. The KMO test value of the questionnaire is 0.670, which is greater than 0.6. Therefore, the null hypothesis of Bartlett's test is rejected, showing that the questionnaire has good validity.

### 4.3. The Difference before and after the Experiment

#### 4.3.1. Variances among Elements of the Experimental Group

Figure 6 shows the differences in the test results before and after the investigation.

Figure 6 shows that the standard deviation of students' learning attitudes to IPE is 0.98, and the average is 2.74 in the pretest of the experimental group. After big data introduction, the standard deviation of the educated is 1.07, with an average of 2.97. The standard deviation of students' participation is 0.6, with an average of 2.96. The average recognition of teaching effect is 2.86, and its standard deviation is 1.02. The average value of students' understanding and recognition of the IPE learning content is 3.02, and its standard deviation is 0.95. The average value of the teaching situation on the learning effect of IPE is 3.15, and its standard deviation is 1.22. The teaching content of IPE is 3.23, and its standard deviation is 1.25.

In summary, the mean values of teaching content, mastery and recognition of IPE knowledge, and teaching situation are all higher than 3, and the mean values of their influencing factors are lower than 3. Therefore, the scores of various influencing factors in the pretest are low. The *T*-values of the mastery and recognition of teaching content is −2.256, and its visibility is 0.026, less than 0.05. The *T*-value of the educated is −2.334, and its visibility is 0.021, less than 0.05. The *T*-value of educators is −4.199, and its significance is 0.000, less than 0.05. The *T*-value of students' attitudes towards IPE is −3.108, and its visibility is 0.002, less than 0.05. The *T*-value of teaching content is −2.527, and its significance is 0.013, less than 0.05. The *T*-value of the teaching situation is −2.656, and its obviousness is 0.009, less than 0.05. The *T*-value of students' recognition of the teaching effect is −2.384, and its obviousness is 0.019, less than 0.05. Therefore, it is concluded that the influencing factors show noticeable differences after two tests. The scores of each influencing factor in the posttest process are higher than those in the pretest, indicating that big data can improve students' learning effects of IPE.

#### 4.3.2. Variances among Elements of the Control Group

Figure 7 shows the difference of each influencing factor in the control group.

Figure 7 shows that the *T*-value of students' recognition of the teaching effect of IPE is −1.742, and its sig. is 0.083, more significant than 0.05. The *T*-value of the teaching content is −0.710, and its sig. is 0.482, more excellent than 0.05. The *T*-value of students' mastery and recognition of the knowledge is −1.091, and its sig. is 0.266, more significant than 0.05. The *T*-value of the teaching situation is −1.246, and its sig. is 0.215, more significant than 0.05. The *T*-value of the educated is −0.408, and its sig. is 0.684, more significant than 0.05. The *T*-value of students' learning attitudes is −0.897, and its sig. is 0.371, more significant than 0.05. The *T*-value of educators is −0.919, and its sig. is 0.360, greater than 0.05. The students' values in the control group in the posttest are the same as those in the pretest. In contrast, the students' values in the experimental group in the posttest are significantly improved. It indicates that big data has a significant impact on improving the teaching quality of IPE.

## 5. Discussion

Compared with the traditional teaching mode of IPE, the teaching mode based on big data has the following advantages:

1. The introduction of big data into IPE can give students “new channels” to receive IPE and enhance their overall identity. Generally, identity refers to students' positive emotions and evaluations of IPE. However, according to the survey results, more than 50% of college students have an indifferent attitude towards identity. They believe that they receive IPE only to pass the examination, limiting their IPE cognition. Based on identity, students can participate in IPE actively and are willing to combine their original ideological and cognitive basis with the content of IPE, realizing internal moral constraints and external behavioral support.
2. It can help update the teaching methods and improve students' autonomous learning ability. It is similar to MOOCs and Yiban virtual campus based on the application of Internet teaching platform and enriches the diversity of teaching methods. The main channel for IPE is the classroom teaching of ideological and political theories, but its actual effect differs from person to person. The real feelings generated by students in the learning process are partly based on their attitudes and partly derived from the personal perception under the external influence factors. Although there are sampling questions or typical examples, it is not clear whether the overall effect is improved and whether students' learning autonomy is improved. Besides, applying various teaching platforms and information-based teaching methods can bring multiple changes. It can witness students' ideological changes and achievements. The Internet's convenient, fast, and independent operation encourages students to consciously participate in the selection, learning, and feedback, which provides a reference for the following teaching period.
3. It can provide data-based evaluation for IPE. A crucial advantage of big data is that “everything can be quantified.” All subjective, objective, abstract, and complex information can be converted into quantifiable data. The influence of digital information on the classroom teaching of IPE is not exceptional. Students' scores, credit points, attendance rate, and head-raising rate can be quantified, and the data or graphics can show their real states. Data are not everything, but there is no basis for its evaluation stage without data. The openness of the Internet dramatically increases the acquisition rate of data, and all aspects of students' learning and life are “traceable.” Whether they are texts, pictures, audios, or videos, the data can be filtered and purified through inductive analysis, becoming a piece of guiding information with a high utilization rate. In addition, the changing trend of students' attitudes is the same as that of people's electrocardiogram, showing different curves or forms under the influence of influencing factors. However, people's psychological internalization is essentially a complex and changeable process. Under the visual analysis of data, the attitude change model can be implemented, and quantitative and evaluation data can be obtained.

## 6. Conclusions

The influence of big data on college students' learning effects of IPE under AI is discussed. Big data is introduced into the classroom teaching of IPE after its characteristics are analyzed. The influence of big data on teaching quality is explored in the experimental and control groups. The results show that the students in the experimental group achieve better learning effects. They have good performance in the mastery and recognition of learning content and the teaching effect. It shows that, in the AI era, big data can help college students better grasp the teaching content of IPE, and their learning enthusiasm is incredibly inspired. However, the study also has some limitations. Big data is not mature, so they are not applied universally. It needs to be explored and discussed further. This work provides a reference for the follow-up study, hoping that more technologies can be used in classroom teaching with the progress of science and technology.

## Figures and Tables

**Figure 1:** Features of big data.

**Figure 2:** Data-driven decision-making structure of big data.

**Figure 3:** Gender statistics (A: male students; B: female students; C: total number).

**Figure 4:** Statistics of political outlook (A: members of communist party of China (CPC); B: members of the communist youth league; C: the masses; D: total).

**Figure 5:** Elements of improving the teaching quality of IPE (A: teaching methods and content; B: students' enthusiasm; C: teaching atmosphere; D: testing form).

**Figure 6:** Differences of the influencing factors in the experimental group (A: learning attitudes; B: the educated; C: educators; D: teaching content; E: teaching situation; F: mastery and recognition of the learning content; G: understanding and recognition of learning content).

**Figure 7:** Differences of each factor in the control group (A: learning attitudes; B: the educated; C: educators; D: teaching content; E: teaching situation; F: mastery and recognition of the knowledge; G: recognition of the teaching effect of IPE).

**Table 1:** Statistics of influencing factors of teaching effectiveness.

	Number of people	Percentage	Effective percentage
Student attitude	80	33.3	33.3
Teacher's teaching method	68	28.3	28.3
Learning atmosphere	35	14.6	14.6
Course content	57	23.8	23.8

**Table 2:** Statistics of reliability test results of the questionnaire.

Dimension	Number of items	Cronbach's alpha
A	3	0.799
B	3	0.793
C	3	0.858
D	3	0.927
E	3	0.865
F	5	0.863
G	4	0.782

A: learning attitude; B: educatee factor; C: educator factor; D: teaching information factor; E: teaching situation factor; F: mastery and recognition of learning content; G: understanding and recognition of learning content.

**Table 3:** Statistics of validity results.

KMO		0.67
Bartlett	A	1404.359
	B	253
	C	0.000

A: approx. chi-square; B: degree of freedom (df); C: significant level (sig.).

## Data Availability

The data used to support the findings of this study are available from the corresponding author upon request.
